# Application of Different Doses of Dexmedetomidine Combined with General Anesthesia in Anesthesia of Patients with Traumatic Tibiofibular Fractures and Its Effect on the Incidence of Adverse Reactions

**DOI:** 10.1155/2021/3080098

**Published:** 2021-12-14

**Authors:** Jizheng Zhang, Xiaohua Sun, Wenjie Cheng, Wanlu Ren

**Affiliations:** Department of Anesthesiology, Outpatient and Emergency,Tianjin Hospital, Tianjin 300211, China

## Abstract

**Objective:**

To explore the application of different doses of dexmedetomidine combined with general anesthesia in patients with traumatic tibiofibular fractures.

**Methods:**

A total of 120 patients with traumatic tibiofibular fractures treated in our hospital (January 2018–January 2021) were selected as the research subjects and equally grouped into group A, group B, group C, and group D according to the dosage of dexmedetomidine. Group B, group C, and group D were pumped with 0.3 *μ*g/kg, 0.5 *μ*g/kg, and 0.8 *μ*g/kg load doses of dexmedetomidine before anesthesia induction, with the same doses for maintenance during surgery. Group A was intravenously pumped with the same amount of normal saline and received tracheal intubation after anesthesia induction, with propofol and remifentanil to maintain general anesthesia during surgery.

**Results:**

No notable differences in general data were observed among the groups (*P* > 0.05). Ramsay sedation scores of all groups showed a downward trend after drug withdrawal. At 10 min, 30 min, and 60 min, the scores of groups *C* and *D* were markedly higher than those of groups A and B (*P* < 0.05), and the scores were higher in group D than those in group C (*P* < 0.05). The HR changes at each period were close between groups A and B (*P* > 0.05). The HRs at T1 and T2 in group C were slightly lower than those in group D (*P* > 0.05), and the HRs at T1 in groups A and B were remarkably higher than those in groups C and D, and were higher than those at T0 and T2 (*P* < 0.05). The SBP levels of all groups began to rise at T0, peaked at T1, and decreased to a lower level at T2 than that at T0. Moreover, the SBP levels of groups C and D at T1 and T2 were notably lower compared with groups A and B (*P* < 0.05). With a lower DBP level in group C than the other three groups at T1, the DBP levels were notably lower in groups C and D than those in groups A and B at T2 (*P* < 0.05). With no statistical difference in the MAP levels at T0 among the four groups (*P* > 0.05), the MAP levels in group A at T1 and T2 were obviously higher compared with groups C and D (*P* < 0.05). The extubation time in group A was notably longer than that that in groups B, C, and D (*P* < 0.05), with longer extubation time in group B than that in groups C and D (*P* < 0.05). The orientation recovery time in group D was markedly shorter than that in groups A, B, and C (*P* < 0.05). The incidence of cognitive dysfunction, chills, and restlessness in groups C and D was notably lower compared with groups A and B (*P* < 0.05), with a higher incidence of chills, intraoperative hypotension, and delayed awakening in group D than in group C (*P* < 0.05).

**Conclusion:**

Dexmedetomidine at doses of 0.5 *μ*g/kg and 0.8 *μ*g/kg has a better effect in the maintenance of general anesthesia for patients with traumatic tibiofibular fractures, with faster orientation recovery, better recovery of postoperative cognitive function, and a lower incidence of adverse reactions. Dexmedetomidine at 0.5 *μ*g/kg is recommended in view of the increased risk of excessive sedation, chills, restlessness, and intraoperative hypotension in patients at 0.8 *μ*g/kg.

## 1. Introduction

Tibiofibula is the most vulnerable part of long tubular bones, with the fracture rate accounting for about 13.7% of the whole body. Tibiofibular fractures are mostly caused by direct or indirect violence, and the patients suffer from pain, swelling, local deformity, and even dysfunction in the fracture sites [1–3]. At present, surgical reduction and fixation is the main method for treating traumatic tibiofibular fractures, which can easily lead to skin damage due to less subcutaneous tissue on the anteromedial side of the tibia and can easily induce the post-traumatic stress response in patients due to the large trauma of surgery, aggravating the inflammatory degree of the body and hindering the healing of the fractures. However, scientific and reasonable anesthesia in surgery can help patients maintain homeostasis and reduce stress response, and it has been reported that the intraoperative anesthesia effect is closely related to the amount of anesthetic. Dexmedetomidine, a selective *α*2-adrenoceptor agonist with short half-life, has sedative and analgesic effects, inhibits sympathetic nerve activity, attenuates the stress response to tracheal intubation, and stabilizes hemodynamics, which is widely adopted to assist in general anesthesia [4–6]. Suitable dosage of anesthetic can directly affect patients' recovery after surgery. However, there is some controversy about the reasonable dose of dexmedetomidine for general anesthesia at present, and its application in reduction and fixation of traumatic tibiofibular fractures is rarely reported. Therefore, this study will explore the effect of different doses of dexmedetomidine combined with general anesthesia on awakening quality, hemodynamics, and adverse reactions of patients undergoing reduction and fixation of traumatic tibiofibular fractures.

## 2. Study Protocol

### 2.1. Case Selection and Grouping

One hundred and twenty patients with traumatic tibiofibular fractures treated in our hospital (January 2018–January 2021) were selected as the research subjects and equally grouped into group A, group B, group C, and group *D* according to the dosage of dexmedetomidine. The study was approved and supervised by the hospital ethics committee.

### 2.2. Inclusion Criteria

The following are the inclusion criteria: (1) the patients met the clinical diagnostic criteria for traumatic tibiofibular fractures established by the Chinese Medical Association [7], with the surgical indications of general anesthesia; (2) the patients had high treatment compliance and complete follow-up; (3) the patients had no history of drug allergy used by the study; (4) the patients' chief complaint was clear; (5) the patients did not have other somatic diseases; and (6) both patients and family members were informed of this study.

### 2.3. Exclusion Criteria

The following are the exclusion criteria: (1) the patients complicated with other diseases affecting ankle function; (2) the patients complicated with malignancies, hypertension, diabetes mellitus, and chronic liver and kidney diseases; (3) the patients with cognitive impairment or communication disorders; (4) pregnant and lactating women; and (5) the patients who did not have complete medical records.

### 2.4. Methods

The patients were fasted and deprived of water for 8 hours before surgery. After entering the operating room, the venous channel was opened. Electrocardiograph (ECG), heart rate (HR), and blood oxygen saturation (SpO_2_) were closely monitored, and invasive blood pressure monitoring was established under local anesthesia [8–10]. Dexmedetomidine was diluted to 4 *μ*g/mL; 0.01 mg/kg of penehyclidine was intravenously injected at 30 min before anesthesia induction. Group *B*, group *C,* and group *D* were pumped with 0.3 *μ*g/kg, 0.5 *μ*g/kg, and 0.8 *μ*g/kg load doses of dexmedetomidine at 15 min before anesthesia induction, with the same doses for maintenance during surgery. Group A was intravenously pumped with the same amount of normal saline. Anesthesia induction was carried out as follows. After mask oxygen inspiration for 3 min, the patients were intravenously injected with 0.1 mg/kg of midazolam, 4 *μ*g/kg of fentanyl, 5 *μ*g/mL of propofol, and 0.15 mg/kg of cisatracurium. After induction, tracheal intubation was performed by the same anesthetist. Propofol (5 mg/kg·h) and remifentanil (0.2 *μ*g/kg·min) were micropumped to maintain intraoperative general anesthesia, and cisatracurium was given according to the actual situation of the patients. Additional intravenous anesthetics were stopped at 30 min before the end of surgery, and the pumping of dexmedetomidine was stopped before suturing [11–13]. The secretions in the catheter and oral cavity were aspirated at the end of the surgery. When the patients were conscious, and coughing, with the recovery of swallowing reflex, spontaneous breathing, and SpO_2_ (more than 97%), the tracheal tube was removed. Routine postoperative analgesia was performed [14].

### 2.5. Observation Indexes

The age, BMI, interval between fracture and surgery, gender, AO classification of fractures, and causes of injury were recorded. The Ramsay sedation score was used to evaluate the sedation degree of patients at 10 min, 30 min, and 60 min after the withdrawal of anesthetics, which was divided into 1 point (nervousness and restlessness), 2 points (quietness, orientation, and cooperation), 3 points (following instructions and drowsiness), 4 points (patients who could be awakened), 5 points (slow breathing and response), and 6 points (patients who were in deep sleep and could not be awakened).

The hemodynamic indexes were measured at the end of surgery (T0), extubation (T1), and 5 min after extubation (T2), mainly including heart rate (HR), systolic blood pressure (SBP), diastolic blood pressure (DBP), and mean arterial pressure (MAP). The orientation recovery time, extubation time, and perioperative adverse reactions were recorded.

### 2.6. Statistical Treatment

The data were statistically processed by SPSS 22.0 software and graphed by GraphPad Prism 7 (GraphPad Software, San Diego, USA). The data included enumeration data and measurement data, expressed as (*n* (%)) and (‾*x* ± *s*) and tested by the *X*^2^ test and *t*-test. The differences were statistically different at *P* < 0.05.

## 3. Results

### 3.1. General Data

The general data such as age, BMI, interval between fracture and surgery, gender, AO classification of fractures, and causes of injury in the four groups were statistically analyzed, and no notable differences in general data were observed among the groups (*P* > 0.05; Table 1).

### 3.2. Ramsay Sedation Scores

Ramsay sedation scores of all groups showed a downward trend after drug withdrawal. At 10 min, 30 min, and 60 min, the scores of groups *C* and *D* were markedly higher than those of groups A and B (*P* < 0.05), and the scores were higher in group *D* than in group C (*P* < 0.05; Table 2).

### 3.3. HRs

The HR changes at each period were close between groups *A* and *B* (*P* > 0.05). The HRs at T1 and T2 in group C were slightly lower than those in group *D*, with no statistical difference (*P* > 0.05), and the HRs at T1 in groups A and B were remarkably higher than those in groups C and *D* and were higher than those at T0 and T2 (*P* < 0.05), as presented in Figure 1.

### 3.4. SBP

The SBP levels of all groups began to rise at T0, peaked at T1, and decreased to a lower level at T2 than at T0. Moreover, the levels of groups *C* and *D* at T1 and T2 were notably lower compared with groups A and B (*P* < 0.05; Figure 2).

### 3.5. DBP

With a lower DBP level in group *C* than the other three groups at *T*1, the DBP levels were notably lower in groups *C* and *D* than in groups *A* and *B* at T2 (*P* < 0.05; Figure 3).

### 3.6. MAP

With no statistical difference in the MAP levels at T0 among the four groups (*P* > 0.05), the MAP levels in group A at T1 and T2 were obviously higher compared with groups C and *D* (*P* < 0.05; Figure 4).

### 3.7. Orientation Recovery Time and Extubation Time

The extubation time in group A was notably longer than that in groups *B*, *C,* and *D* (*P* < 0.05), with longer extubation time in group B than that in groups C and *D* (*P* < 0.05). The orientation recovery time in group *D* was markedly shorter than that in groups A, B, and C (*P* < 0.05; Table 3).

### 3.8. Adverse Reactions

The incidence of cognitive dysfunction, chills, and restlessness in groups C and *D* was notably lower compared with groups A and B (*P* < 0.05), with a higher incidence of chills, intraoperative hypotension, and delayed awakening in group *D* than those in group C (*P* < 0.05). No obvious differences in nausea and vomiting and bucking were observed among the four groups (*P* > 0.05). The results are presented in Table 4.

## 4. Discussion

Tibiofibula is a key bone supporting human weight, and its fractures can seriously affect the patients' lower extremity function, especially the ankle function. At present, surgical open reduction is the main method in clinical treatment to promote fracture healing and improve the joint function. However, due to the common peroneal nerve and abundant tissue and blood vessels around the tibiofibula, as well as the large trauma, surgery can easily damage the blood vessels and nerves and induce post-traumatic stress response, accompanied by various postoperative adverse reactions after surgery [15–17]. In addition, patients under general anesthesia experience hemodynamic changes such as increased heart rate and blood pressure due to sympathetic excitation caused by surgical pain and other stimuli as the anesthesia gradually subsides. A number of related studies combined with clinical practice show that dexmedetomidine as an *α*2-adrenoceptor agonist can inhibit the release of adrenaline and acetylcholine by modulating *α*2 adrenoceptors and reduce the cAMP level in cells by decreasing the release of substance P in the presynaptic membrane, thus playing an analgesic and sedative role and maintaining body homeostasis during general anesthesia [18, 19]. At present, the specifically used dose of dexmedetomidine for general anesthesia has not been determined, and there are few related studies, but most of them suggest that it is appropriate to maintain the dosage at 0.2–1.0 *μ*g/kg [20].

In this study, Ramsay sedation scores of all groups showed a downward trend after drug withdrawal. At 10 min, 30 min, and 60 min, the scores of groups C and *D* were markedly higher than those of groups A and B (*P* < 0.05), and the scores were higher in group *D* than in group *C* (*P* < 0.05). The results suggested that most of the patients in group *D* were in deep sleep and had delayed awakening, which might be related to the dose-dependent sedation effect of dexmedetomidine. Small doses will lead to a poor sedation effect, whereas large doses will easily produce excessive sedation and delayed awakening. The HR changes at each period were close between groups A and B (*P* > 0.05). The HRs at *T*1 and *T*2 in group *C* were slightly lower than those in group *D* (*P* > 0.05), and the HRs at T1 in groups A and B were remarkably higher than those in groups *C* and *D*, and were higher than those at T0 and T2 (*P* < 0.05). The SBP levels of all groups began to rise at T0, peaked at T1, and decreased to a lower level at T2 than at T0. Moreover, the SBP levels of groups C and *D* at T1 and T2 were notably lower compared with groups *A* and *B* (*P* < 0.05). With a lower DBP level in group C than the other three groups at T1, the DBP levels were notably lower in groups C and *D* than in groups A and B at T2 (*P* < 0.05). With no statistical difference in the MAP levels at T0 among the four groups (*P* > 0.05), the MAP levels in group A at T1 and T2 were obviously higher compared with groups C and *D* (*P* < 0.05). Summary analysis of the above results shows that dexmedetomidine for general anesthesia at doses of 0.5 *μ*g/kg and 0.8 *μ*g/kg can ensure the stability of hemodynamic indexes in patients undergoing reduction of traumatic tibiofibular fractures. Besides, 0.5 *μ*g/kg dose of dexmedetomidine has less fluctuation of hemodynamic indexes in patients compared with 0.8 *μ*g/kg. The extubation time in group *A* was notably longer than that in groups *B*, *C,* and *D* (*P* < 0.05), with longer extubation time in group B than that in groups *C* and *D* (*P* < 0.05). The orientation recovery time in group *D* was markedly shorter than that in groups *A*, *B,* and *C* (*P* < 0.05). These results are similar to those in the studies of Jehan Ahmed Sayed et al. [21] and Chiara Adami et al. [22], indicating that dexmedetomidine at doses of 0.5 *μ*g/kg and 0.8 *μ*g/kg is notably better than 0.3 *μ*g/kg in promoting orientation recovery of patients. In addition, the incidence of cognitive dysfunction, chills, and restlessness in groups C and *D* was notably lower compared with groups *A* and *B* (*P* < 0.05), with a higher incidence of chills, intraoperative hypotension, and delayed awakening in group *D* than in group *C* (*P* < 0.05). It could be concluded that the patients in group C had the lowest incidence of chills, intraoperative hypotension, and delayed awakening among the four groups, with no statistical differences in the cognitive dysfunction and restlessness between groups C and D. The reasons are as follows. (1) Hypotension and hypothermia are the main causes of chills during the recovery period of general anesthesia. Dexmedetomidine can prevent chills by the inhibition of potassium ion influx, obvious cell depolarization, and low sensitivity of body temperature regulation system, so the body temperature does not decrease sharply. Moreover, the risk of chills with the addition of dexmedetomidine is lower than that with a lower dose. Hypotension can often be prevented as long as the drug can play a better sedative effect. (2) There is a certain critical value for the sedation effect of dexmedetomidine in sleep time of nonrapid eye movements, and a higher dose exceeding the critical value may lead to excess sedation, thus triggering symptoms such as delayed awakening, hypothermia, and muscle vibration. (3) Low-dose dexmedetomidine has insignificant effect on protecting brain, and both medium and large doses can protect brain function, whereas excessive doses cannot improve the effect of brain protection, but triggers intraoperative hypotension [23–25].

In conclusion, dexmedetomidine at doses of 0.5 *μ*g/kg and 0.8 *μ*g/kg has a good effect in the maintenance of general anesthesia for patients with traumatic tibiofibular fractures, with faster orientation recovery, better recovery of postoperative cognitive function, and a lower incidence of adverse reactions. Dexmedetomidine at 0.5 *μ*g/kg is recommended in view of the increased risk of excessive sedation, chills, restlessness, and intraoperative hypotension in patients at 0.8 *μ*g/kg. The study had a smaller sample size because only 30 patients were enrolled in each group, and it was a single-center study. Subsequently, relevant multicenter studies with an expanded sample size should be carried out to further confirm the correctness of the conclusion.

## Figures and Tables

**Figure 1:** Statistical treatment of HR (‾*x* ± *s*). Note: the abscissa represents the time points, and the ordinate represents the detection level (times/min). The HRs of group A at T0, T1, and T2 were (63.42 ± 3.83), (80.03 ± 5.01), and (70.20 ± 2.14). The HRs of group B at T0, T1, and T2 were (63.35 ± 3.85), (79.84 ± 4.96), and (68.85 ± 2.21). The HRs of group C at T0, T1, and T2 were (63.47 ± 3.82), (68.62 ± 3.78), and (66.97 ± 3.54). The HRs of group D at T0, T1, and T2 were (63.15 ± 4.23), (70.03 ± 5.15), and (67.44 ± 3.52). ^*∗*^The HRs at T1 in groups A and B were notably higher than those in groups C and *D* (*P* < 0.05); ^*∗∗*^the HRs at T1 in groups A and B were notably higher than those at T0 (*P* < 0.05); ^*∗∗∗*^the HRs at T1 in groups A and B were notably higher than those at T2 (*P* < 0.05).

**Figure 2:** Statistical treatment of SBP (‾*x* ± *s*). Note: the abscissa represents the time points, and the ordinate represents the detection level (mmHg). The SBP levels of group A at T0, T1, and T2 were (124.72 ± 3.95), (134.08 ± 5.31), and (120.88 ± 4.30). The SBP levels of group B at T0, T1, and T2 were (123.50 ± 3.82), (131.49 ± 5.85), and (119.26 ± 4.18). The SBP levels of group C at T0, T1, and T2 were (121.55 ± 3.62), (123.05 ± 5.71), and (114.22 ± 8.29). The SBP levels of group *D* at T0, T1, and T2 were (122.34 ± 3.71), (127.88 ± 6.46), and (113.27 ± 4.46).

**Figure 3:** Statistical treatment of DBP (‾*x* ± *s*). Note: the abscissa represents the time points, and the ordinate represents the detection level (mmHg). The DBP levels of group A at T0, T1, and T2 were (67.11 ± 5.28), (74.89 ± 6.25), and (67.67 ± 5.31). The DBP levels of group B at T0, T1, and T2 were (66.46 ± 5.07), (72.21 ± 6.33), and (68.25 ± 6.44). The DBP levels of group C at T0, T1, and T2 were (66.37 ± 5.14), (72.18 ± 6.29), and (68.10 ± 6.29). The DBP levels of group *D* at T0, T1, and T2 were (66.25 ± 5.10), (72.15 ± 6.33), and (68.11 ± 6.14).  ^*∗*^The DBP level of group C at T1 was remarkably different from that of groups A, B and C (*P* < 0.05).  ^*∗*^ ^*∗*^The DBP levels of groups C and *D* at T2 were obviously different from those of groups *A* and *B* (*P* < 0.05).

**Figure 4:** Statistical treatment of MAP (‾*x* ± *s*). Note: the abscissa represents the time points, and the ordinate represents the detection level (mmHg). The MAP levels of group A at T0, T1, and T2 were (88.25 ± 5.28), (98.39 ± 6.12), and (91.96 ± 5.41). The MAP levels of group B at T0, T1, and T2 were (87.17 ± 5.32), (93.05 ± 5.12), and (88.65 ± 4.63). The MAP levels of group C at T0, T1, and T2 were (87.11 ± 5.16), (90.07 ± 4.86), and (87.09 ± 4.50). The MAP levels of group *D* at T0, T1, and T2 were (87.59 ± 5.43), (91.25 ± 6.15), and (88.04 ± 5.13). ^*∗*^The MAP level of group A at T1 was notably higher than that of groups *B*, *C,* and *D* (*P* < 0.05). ^*∗∗*^The MAP level of group A at T2 was notably higher than that of groups *B*, *C,* and *D* (*P* < 0.05).

**Table 1:** Statistical treatment of general data (*n* = 30).

Observation indexes	Group A	Group B	Group C	Group D
Age	41.85 ± 3.74	40.92 ± 4.06	42.11 ± 3.89	41.68 ± 3.77
BMI (kg/m^2^)	25.84 ± 3.26	26.15 ± 3.31	25.74 ± 3.50	26.09 ± 3.43
Interval between fracture and surgery (h)	7.37 ± 2.86	7.55 ± 3.22	7.64 ± 3.18	7.42 ± 3.05

*AO classification of fractures*				
A	13 (43.33)	15 (50)	12 (40)	14 (46.67)
B	12 (40)	12 (40)	13 (43.33)	11 (36.67)
C	5 (16.67)	3 (10)	5 (16.67)	5 (16.67)

*Gender*				
Male	14 (46.67)	12 (40)	15 (50)	16 (53.33)
Female	16 (53.33)	18 (60)	15 (50)	14 (46.67)

*Causes of injury*				
Accidents	12 (40)	13 (43.33)	15 (50)	13 (43.33)
Falls	12 (40)	13 (43.33)	12 (40)	11 (36.67)
Crushing from heavy loads	6 (20)	4 (13.33)	3 (10)	6 (20)

Note. Under various dimensions, the statistical differences in general data among groups A, B, C, and D were not significant (*P* > 0.05).

**Table 2:** Statistical treatment of Ramsay scores (‾*x* ± *s*).

Group	*n*	10 min	30 min	60 min
*A*	30	3.21 ± 0.88	2.88 ± 0.39	2.41 ± 0.55
*B*	30	3.35 ± 0.80	3.03 ± 0.54	2.38 ± 0.47
*C*	30	4.02 ± 0.75^*∗*^b	3.28 ± 0.38^*∗*^b	3.02 ± 0.45^*∗*^b
*D*	30	4.38 ± 0.61^*∗*^bc	4.05 ± 0.45^*∗*^bc	3.36 ± 0.55^*∗*^bc

*Note*. ^*∗*^*P* < 0.05, compared with group A; *bP* < 0.05, compared with group B; *cP* < 0.05, compared with group *C*.

**Table 3:** Statistical treatment of orientation recovery time and extubation time (‾*x* ± *s*).

Group	*n*	Extubation time (min)	Orientation recovery time (min)
*A*	30	21.89 ± 1.07	25.94 ± 2.01
*B*	30	19.37 ± 1.96^*∗*^	22.64 ± 2.78^*∗*^
*C*	30	18.20 ± 1.20^*∗*^b	22.02 ± 2.60^*∗*^
*D*	30	17.71 ± 1.68^*∗*^b	10.05 ± 2.10^*∗*^bc

*Note*.  ^*∗*^*P* < 0.05, compared with group A; *b* *P* < 0.05, compared with group B; *c* *P* < 0.05, compared with group C.

**Table 4:** Statistical treatment of incidence of adverse reactions (n (%)).

Group	Cognitive dysfunction	Chills	Restlessness	Intraoperative hypotension	Nausea and vomiting	Delayed awakening	Bucking
*A*	14 (46.67)	12 (40)	6 (20)	1 (3.33)	3 (10)	0 (0)	4 (13.33)
*B*	12 (40)	11 (36.67)	6 (20)	1 (3.33)	2 (6.67)	0 (0)	2 (6.67)
*C*	5 (16.67)^*∗*^b	0 (0)^*∗*^b	1 (3.33)^*∗*^b	1 (3.33)	3 (10)	1 (3.33)	2 (6.67)
*D*	4 (13.33)^*∗*^b	4 (13.33)^*∗*^bc	1 (3.33)^*∗*^b	6 (20)^*∗*^bc	3 (10)	6 (20)^*∗*^bc	3 (10)

*Note*. ^*∗*^*P* < 0.05, compared with group A; *b* *P* < 0.05, compared with group B; *c* *P* < 0.05, compared with group C.

## Data Availability

Data to support the findings of this study are available on reasonable request from the corresponding author.
